The article "Development of cellulose-based conductive fabrics with electrical conductivity and flexibility" was published in 2020. Journal: PLoS One.

# Development of cellulose-based conductive fabrics with electrical conductivity and flexibility

**DOI:** 10.1371/journal.pone.0233952

**Published:** 2020-06-04

**Authors:** Hyunjin Kim, Joon-Yeop Yi, Byung-Gee Kim, Ji Eun Song, Hee-Jin Jeong, Hye Rim Kim

**Affiliations:** 1 Department of Clothing and Textiles, Sookmyung Women's University, Seoul, South Korea; 2 Interdisciplinary Program of Bioengineering, Seoul National University, Seoul, South Korea; 3 Institute of Molecular Biology and Genetics, Seoul National University, Seoul, South Korea; 4 School of Chemical and Biological Engineering, Seoul National University, Seoul, South Korea; 5 Human Convergence Technology Group, Korea Institute of Industrial Technology, Ansan, South Korea; 6 Department of Biological and Chemical Engineering, Hongik University, Sejong, South Korea; University of Maryland Baltimore County, UNITED STATES

## Abstract

This study aimed to produce cellulose-based conductive fabrics with electrical conductivity and flexibility. Bacterial cellulose (BC) and three chemical cellulose (CC), namely methyl cellulose (MC), hydroxypropyl cellulose (HPMC) and carboxymethyl cellulose (CMC) were *in situ* polymerized with aniline and the four conductive cellulose fabrics were compared and evaluated. Matrix-assisted laser desorption/ionization time-of-flight mass spectroscopy analysis confirmed that three CC-PANI composites displayed longer and more stable polymerization pattern than BC-PANI because of the different polymerization method: bulk polymerization for BC-PANI and emulsion polymerization for CC-PANI, respectively. The electrical conductivity of BC-PANI and CC-PANI were ranging from 0.962 × 10^−2^ S/cm to 2.840 × 10^−2^ S/cm. MC-PANI showed the highest electrical conductivity among the four conductive cellulose fabrics. The flexibility and crease recovery results showed that MC-PANI had the highest flexibility compared to BC-PANI, HPMC-PANI, and CMC-PANI. These results have confirmed that the electrical conductivity and flexibility were influenced by the type of cellulose, and MC-PANI was found to have the best performance in the electrical conductivity and flexibility.

## Introduction

Conductive fabrics are electrically functionalized fabrics with the advantages of flexibility, elasticity, and wearability [1, 2]. These features have enabled conductive fabrics to be applied for textile-integrated batteries [3], wearable sensors [4], and fabric-based energy storage devices [5]. Conductive fabrics can be manufactured by the weaving and knitting of conductive threads [6] or by synthesizing conductive polymers onto the fabric material [7]. The synthesis method is commonly used because of the simple manufacturing process [8]. Conductive polymers, such as polypyrrole, polyaniline, and polythiophene, are organic-based polymers with extended π-orbital systems along their conjugate backbone through which electrons can move freely [9]. Due to their unique structure, conductive polymers are lighter and better resist corrosion than metals [10].

The article "Development of cellulose-based conductive fabrics with electrical conductivity and flexibility" was published in 2020. Journal: PLoS One.

Among the various conductive polymers, polyaniline (PANI) has been widely studied because of its good chemical stability, good electrical conductivity, and ease of synthesis by the *in situ* polymerization of aniline [11–13]. In this study, PANI was polymerized onto cellulose to produce the conductive fabric. However, PANI has poor mechanical properties since it is inherently very stiff [14]. To overcome the disadvantage of PANI, a flexible fiber material is required to be synthesized with PANI [15].

Cellulose is one of the most abundant natural fibers. It is composed of glucose chains that contain many hydroxyl (-OH) functional groups [16]. It has excellent physical properties, such as flexibility, and is biodegradable [17]. Because of these properties, cellulose is considered as a good material to produce conductive fabrics. The characteristics of cellulose vary depending on its origin [18]. Presently, bacterial cellulose (BC) and chemical cellulose (CC), especially methyl cellulose (MC), carboxymethyl cellulose (CMC), and hydroxypropyl methyl cellulose (HPMC) were used. BC is produced *Acetobacter xylinus* bacteria. BC has a three-dimensional nanostructure with pronounced biocompatibility and purity [19, 20]. MC is derived from chemical cellulose without loss of biocompatibility [21]. It is formed by replacing the hydroxyl groups of cellulose with methoxy groups through chemical modification to improve the water solubility of cellulose [22]. The ease of water-based MC modification suggests the possibility of wet spinning and ink material produced by three-dimensional printers. Other advantages of MC include transparency, elasticity, and mechanical strength [22]. Also. HPMC and CMC were used to compare those electrical conductivity to the one of MC. These three CC have similar chemical structures but MC has methyl group instead of cellulose hydroxyl groups whereas HPMC has methyl and hydroxyl propyl groups and CMC has carboxymethyl group. HPMC and CMC also have the properties of reasonable biocompatibility, water solubility, transparency and elasticity [23].

Many studies have explored the production of conductive BC-PANI by polymerizing aniline with BC. However, little is known concerning the polymerization of aniline with CC [24, 25]. Moreover, no study has investigated the production of CC-PANI as a conductive fabric, or compared and evaluated BC-PANI and CC-PANI.

The article "Development of cellulose-based conductive fabrics with electrical conductivity and flexibility" was published in 2020. Journal: PLoS One.

The aim of this study is to produce the conductive cellulose fabric with electrical conductivity and flexibility. BC-PANI and three CC-PANI composites are produced, and then compared to select a conductive cellulose fabric with better performance. The polymerization conditions are optimized by ultraviolet-visible (UV-Vis) spectroscopy, and the degree of polymerization is observed with matrix-assisted laser desorption/ionization time-of-flight mass spectroscopy (MALDI-TOF MS). The electrical conductivity, flexibility and crease recovery of conductive cellulose fabrics are evaluated. Chemical and physical structures of conductive cellulose fabrics are evaluated using Fourier-transform infrared spectroscopy (FT-IR) and X-ray diffraction (XRD). Lastly, surface morphology is observed by field-emission scanning electron microscopy (FE-SEM).

## Materials and methods

### Materials

MC powder with a viscosity of 4,000 cP (in 2% solution) and HPMC powder with a viscosity of 4,260 cP (in 2% solution) were obtained from LOTTE Fine Chemical Co., Ltd (Incheon, Korea). CMC sodium salt with a viscosity of 50 to 200 cp (in 4% solution) was obtained from Sigma Chemical CO., (St. Louis, MO, USA). Yeast extract and peptone were purchased from BD Biosciences (San Jose, CA, USA). Glucose, hydrogen peroxide (34.5%), sodium hydroxide, ethyl alcohol (99.9%) and acetic acid were supplied by Duksan Pure Chemical Co., Ltd. (Seoul, Korea). Dodecylbenzene sulfonic acid (DBSA) and trifluoroacetic acid (TFA) were purchased from Sigma-Aldrich (St. Louis, MO, USA). Aniline and acetonitrile were purchased from Junsei Chemical Co., Ltd. (Tokyo, Japan). Ammonium peroxydisulfate (APS) was supplied by Kanto Chemical Co., Inc. (Tokyo, Japan). All chemical reagents were used as received.

### Production of BC-PANI

BC was produced according to a previously reported method [26] and was pre-treated by following the method of Song et al. [27]. Briefly, *Acetobacter xylinus* inoculum was prepared with Hestrin-Schramm (HS) medium (20 g/L glucose, 5 g/L yeast extract, and 5 g/L peptone) and the medium was boiled at 100°C for 10 min. After that, BC was statically cultured at 26°C for 8 days until the thickness of BC became 1 cm. Afterwards, BC was washed with a 3% sodium hydroxide solution at 25°C for 90 min with shaking at 50 rpm, neutralized with distilled water (DW), and adjusted to pH 3.0 using acetic acid for 30 min. After that, BC was bleached with a 5% hydrogen peroxide solution at 90°C for 60 min with shaking at 110 rpm, swelled with an 8% sodium hydroxide solution in a liquor ratio of 1:10 (w/v) for 30 min in an ultrasonic bath, and dried at 35°C.

The article "Development of cellulose-based conductive fabrics with electrical conductivity and flexibility" was published in 2020. Journal: PLoS One.

BC-PANI was produced by the bulk polymerization process by following the method of Kim et al. [28] (Fig 1(A)): First, 2.5 mM aniline and pre-treated BC were added to a 2.5 mM DBSA solution of pH ranging from 2.0 to 4.0. After that, the aniline, BC, and DBSA mixture was magnetically stirred for 1 h. Next, a 2.5 mM APS solution was added to the reaction mixture whereby polymerization was initiated. After several hours at varied temperatures, ranging from 10 to 30°C, BC-PANI was synthesized. The reaction product was washed with an ethanol solution to remove the residue and dried at 25°C for 4 h to produce the nonwoven BC-PANI fabric.

**Fig 1:** Schematic representations of the production process of (A) BC-PANI and (B) CC-PANI, and of (C) bulk polymerization and emulsion polymerization.

### Production of CC-PANI

CC-PANI was produced by the emulsion polymerization process (Fig 1(B)): A solution of 25 mM DBSA was added dropwise into 9 mL of cold DW without mixing to avoid self-micelle formation. After adding 25 mM aniline, the solution was strongly vortexed for 90 sec until its appearance changed to that of a milky white emulsion. The resulting emulsion was incubated for 30 min in an ice bath, and then, polymerization was triggered by adding 1 mL of a 25 mM APS solution. Following a 4-h incubation period, the solution color turned to dark green owing to the formation of the polyaniline-emeraldine salt. At that point, 0.5 g of each CC powder was completely dissolved in 10 mL of the PANI solution. The MC and PANI mixture was transferred to a petri dish and vacuum was applied to remove extra air bubbles, followed by drying at 4°C for 24 h to form the CC-PANI fabric without wrinkling. All chemical components and conical tubes were cooled down before use.

The production of CC-PANI by mixing DBSA, aniline, APS, and CC powder, was optimized with respect to the order of mixing as well as the amount of each component (Fig 1(B)): At first, we confirmed the gelation of the CC powder, necessary to generate sheet-type CC. When we mixed CC powder with DW and heated the mixture for 10 min, solation was observed. After that, we cooled down the sample to room temperature, and confirmed the sol-gel transition. As the hydrogen bonds between MC polymer chains and water molecules were broken at high temperature, the methoxy groups became exposed [23]. Thus, hydrophobic interactions could occur, resulting in the formation of a gel network. Bearing this in mind, we immediately poured the mixture after heating from a glass vial onto a plate, and cooled it down to 4°C, to produce sheet-type CC. Based on this result, we adopted the following procedure: First, we added aniline to DBSA in water and then, mixed the solution with APS. After the color of the solution turned to dark green, we added CC. Finally, we poured the aqueous CC-PANI solution onto a plate and dried it for further characterization.

The article "Development of cellulose-based conductive fabrics with electrical conductivity and flexibility" was published in 2020. Journal: PLoS One.

### UV-Vis spectroscopy

UV spectra of BC- and CC-PANI polymer solutions were acquired with a 96-quartzo microplate reader (SynergyMx, Shimadzu, Japan) for BC-PANI or a cuvette type reader (Thermo Labsystems Multiskan Spectrum, Vantaa, Finland) for CC-PANI, in the absorbance spectrum range from 300 to 800 nm with a resolution of 2 nm. The solutions were diluted 50 times with Milli-Q water before spectrum acquisition.

### MALDI-TOF MS analysis

The polymerization degrees of BC-PANI and CC-PANI were analyzed using a MALDI-TOF/TOF MS 5800 System (AB SCIEX, USA) equipped with a 1 kHz Opti-Beam^TM^ on-axis laser, and a MALDI-TOF Voyager DE-STR (Applied Biosystems, USA) system equipped with a 337-nm nitrogen laser in the linear positive mode, respectively. All samples were dissolved in a TA50 (50% acetonitrile/50% water with 0.1% TFA) solution and mixed with α-cyano-4-hydroxycinnamic acid (CHCA) or 2, 5-dihydroxybenzoic acid (DHB) as a matrix. The samples (0.5 μL) were placed in a 384 Opti-TOF stainless steel plate (AB SCIEX, USA).

### Electrical conductivity

Dried BC- and CC-PANI were split to 1×1 cm pieces, and the thickness of the samples was calculated by using a micrometer (SYNTEK, China). The electrical conductivity of BC- and CC-PANI was measured with the four-point probe method (CMT-SR1000N, Chang Min Tech Co., Ltd., Korea). The electrical resistivity was measured 5 times on different sides and the average was calculated to obtain the surface resistance value. The electrical conductivity was calculated according to the following Eq (1):

$$\sigma =\frac{1}{\left(R\times d\right)}$$ (1)

where σ stands for the electrical conductivity (S/cm), R stands for the electrical resistivity (Ω·cm), and d denotes the thickness of the sample (cm).

### Flexibility and crease recovery test

The flexibility of samples was tested according to KS K 0538 (the heart-loop method) with some modifications. The size of samples was modified to 5 x 10 cm and the experiment time was changed to 1 minute. Samples were made to a loop and after 1 minute, the change in physical properties of samples were compared and evaluated. The crease recovery angles of samples were measured according to KS K 0550 (the recovery angle method). The tests were performed five times for each sample and the results were averaged. The crease recovery was calculated according to the following Eq (2):

$$\mathrm{Crease}\;\mathrm{recovery}\;(\%)=\frac{\mathrm{crease}\;\mathrm{recovery}\;\mathrm{angle}\;({}^{\circ})}{180{}^{\circ}}\times 100$$ (2)

The article "Development of cellulose-based conductive fabrics with electrical conductivity and flexibility" was published in 2020. Journal: PLoS One.

### FT-IR spectroscopy

FT-IR spectra of BC- and CC-PANI were obtained using a Nicolet IS 50 FT/IR spectrophotometer (Thermo Fisher Scientific, Waltham, MA, USA) and TENSOR27 spectrometer (Bruker, Germany), respectively. Scans were acquired between 4,000 cm^-1^ and 650 cm^-1^. The peak resolution was 0.4 cm^-1^ and the number of scans were 32. Baseline correction for each sample spectrum was performed using the Origin 2019 software.

### XRD

The crystalline structure of BC- and CC-PANI were studied with a D8 Advance diffractometer (Bruker AXS Inc., Carlsruhe, Germany) and a X-ray diffractometer (Rigaku, Japan), respectively, using nickel-filtered Cu Kα radiation (λ = 1.54 nm) operating at 40 kV and a filament emission of 40 mA. The scanning rate and step size was 0.01° min^-1^ and 0.1° 2 θ for BC-PANI, and 1° min^-1^ and 0.01° 2 θ for CC-PANI, respectively, and the diffraction patterns were recorded over a range of 2θ angles from 5 to 40°. The baseline for CC-PANI was subtracted using the Origin software with a smoothing factor of 7 and threshold of 0.01.

### SEM

All samples were platinum-coated in an ion sputter prior to the observation. BC-PANI and CC-PANI was imaged using a JSM-7600F microscope (JEOL Ltd., Tokyo, Japan) at 2.0 kV. The PANI sample without BC or MC was imaged at 3.0 kV.

## Results

### Polymerization conditions

The polymerization conditions of BC-PANI and CC-PANI were optimized using UV-Vis spectroscopy. As the PANI polymer solution displays three deterrent colors depending on the oxidation state of PANI, especially green color for PANI emeraldine salt with high electrical conductivity [29], we examined the color change of polymerization solutions of BC-PANI and CC-PANI. UV spectra was observed to determine the optimal point at which PANI was in the emeraldine state. Among three CC-PANI samples, MC-PANI was observed as a representative.

First, the polymerization time was evaluated. As shown in Fig 2, until 0 to 1 h of polymerization, no peak indicative of PANI formation was observed in the UV spectra of both BC-PANI and MC-PANI samples. After 2 h of polymerization for MC-PANI and after 3 h for BC-PANI, the color of the polymer solution changed from white to yellowish-brown, and finally to dark green. Also, the characteristic peaks of PANI were observed in each UV spectrum. In particular, the peaks of PANI corresponded to the π-π* electron transition at 350~360 nm, the polaron- π* transition at 420~430 nm, and the π -polaron transition at 760 nm [30]. This result confirmed that the PANI that had polymerized in BC and CC was in the emeraldine state with good electrical conductivity [29]. Thus, the optimized polymerization time was confirmed as 2 h for CC-PANI and 3 h for BC-PANI. The polymerization time for CC-PANI was shorter than for BC-PANI due to the difference in the polymerization method (Fig 1(C)). Bulk polymerization was used for BC-PANI and emulsion polymerization was used for CC-PANI. As emulsion polymerization is conducted in a controlled micro-scale environment, it has the advantage of being a robust polymerization condition, which reduces the polymerization time. Although we attempted to make an emulsion polymerized BC-PANI, PANI was hardly penetrated to the interior of the BC. As the SEM image showed that BC formed dense fabrics with nanofibers of 100 nm or less in diameter, we thought that the emulsion polymerized PANI particles (10–30 nm in diameter) could not be inserted into the BC. Thus, we performed a bulk polymerization for BC-PANI, which allows aniline monomers to penetrate into tightly woven BC fabrics.

The article "Development of cellulose-based conductive fabrics with electrical conductivity and flexibility" was published in 2020. Journal: PLoS One.

**Fig 2:** The color change and the UV spectra of (A) BC-PANI solution with varied polymerization time from 0 to 3 h, and (B) CC-PANI solution with varied polymerization time from 0 to 2 h.

Other polymerization conditions, such as the molar ratio of DBSA or APS to aniline, the pH level of the DBSA solution, and the polymerization temperature, were evaluated with the same method. The results are summarized in Table 1.

**Table 1:** Polymerization conditions of BC-PANI and CC-PANI.

Polymerization conditions	BC-PANI	CC-PANI
Time	3 hours	2 hours
Molar ratio (DBSA: Aniline)	1.0	1.0
Molar ratio (APS: Aniline)	1.0	1.0
pH level of DBSA solution	pH 2.0	pH 2.0
Temperature	20°C	4°C

### Degree of polymerization

The degree of polymerization (DP) of BC-PANI and CC-PANI was analyzed by MALDI-TOF MS. As shown in Fig 3, consistent peaks of PANI were observed in the mass spectra of BC-PANI and CC-PANI, confirming that PANI was successfully polymerized with BC and CC. In addition, mass intervals of 90 or 91 *m*/*z* appeared in the mass spectra of BC-PANI and CC-PANI, corresponding to the molecular weight of PANI monomer [31]. DP was analyzed according to this interval (Table 2). BC-PANI had short PANI chains with a DP_max_ <5, whereas CC-PANI had longer PANI chains with a DP_max_ of 16 to 17. This result was due to the difference in the polymerization method described in Fig 1(C). The reason why the degree of polymerization rises in an emulsion polymerization is that the emulsion polymerization is based on a radical polymerization, which is occurred with emulsified monomer. Namely, as the concentration of the emulsified monomer in a micelle is high, the interval between the emulsified monomers for mass transfer is shorter than the bulk polymerization [32]. In this study, we used DBSA as a surfactant that traps hydrophobic monomer molecule of aniline into a micelle. But, the monomer molecules of aniline are being dispersed in case of the bulk polymerization. Therefore, the concentration of aniline from emulsion polymerization becomes relatively higher than the one from water-based bulk reaction in the same batch volumes. When the aniline molecules are polymerized, radical molecules around the aniline molecules, such as initiators and activated oligomers, are also being efficiently polymerized, resulting long and stable PANI chains. However, as the aniline monomers are being distributed to the whole container and the distance between aniline monomers in a bulk polymerization are long, the molecules are difficult to reach each other. Thus, the evaluation confirmed that CC-PANI had a more stable polymerization pattern compared to BC-PANI.

The article "Development of cellulose-based conductive fabrics with electrical conductivity and flexibility" was published in 2020. Journal: PLoS One.

**Fig 3:** MALDI-TOF mass spectra of (A)BC-PANI, (B) PANI used in BC-PANI, (C) MC-PANI, (D) HPMC-PANI, (E) CMC-PANI, and (F) PANI used in CC-PANI (polymerization conditions for BC-PANI: pH level of DBSA solution = 2.0, DBSA:aniline:APS = 1:1:1, 20°C, 3 h, polymerization conditions for CC-PANI: pH level of DBSA solution = 2.0, DBSA:aniline:APS = 1:1:1, 4°C, 2 h).

**Table 2:** The degree of polymerization, molecular weight and polydispersity index from mass spectra of PANI, BC-PANI and CC-PANI (polymerization conditions for BC-PANI: pH level of DBSA solution = 2.0, DBSA:aniline:APS = 1:1:1, 20°C, 3 h, polymerization conditions for CC-PANI: pH level of DBSA solution = 2.0, DBSA:aniline:APS = 1:1:1, 4°C, 2 h).

	DP_max_*	Mw **	PDI***
PANI (BC)	5	725.81	1.18
PANI (CC)	12	530.07	1.28
BC-PANI	5	688.30	1.17
MC-PANI	16	948.97	1.18
HPMC-PANI	17	859.08	1.27
CMC-PANI	17	927.58	1.27

*: Maximum degree of polymerization

**: Molecular weight

***: Polydispersity index.

### Electrical conductivity

The thickness and weight of BC- PANI and CC-PANI produced under optimized polymerization conditions were measured, and their electrical conductivity value were 1.990 × 10^−2^ S/cm, 2.840 × 10^−2^ S/cm, 2.080 × 10^−2^ S/cm, and 0.962 × 10^−2^ S/cm, respectively (Table 3). The electrical conductivity measurement indicated that MC-PANI and HPMC-PANI had higher electrical conductivity than BC-PANI, confirming that the electrical conductivity improved as the DP increased due to the formation of long and stable PANI chains.

**Table 3:** Thickness, weight, and electrical conductivity of BC-PANI and CC-PANI (polymerization conditions for BC-PANI: pH level of DBSA solution = 2.0, DBSA:aniline:APS = 1:1:1, 20°C, 3 h, polymerization conditions for CC-PANI: pH level of DBSA solution = 2.0, DBSA:aniline:APS = 1:1:1, 4°C, 2 h).

	Thickness (mm)	Weight (g/m^2^)	Electrical conductivity (S/cm)
BC-PANI	0.218±0.036	138.433±0.273	1.990 × 10^−2^
MC-PANI	0.058±0.007	98.711±0.219	2.840 × 10^−2^
HPMC-PANI	0.052±0.004	84.284±0.472	2.080 x 10^−2^
CMC-PANI	0.080±0.015	103.608±0.398	0.962 x 10^−2^

However, the DP value of CMC-PANI was higher than that of BC-PANI whereas the electrical conductivity of CMC-PANI was lower than of BC-PANI. This can be explained by the differences in the viscosity of cellulose. For conductive polymer composites, it is important how well the polymer is dispersed in the cellulose [33]. If the conductive materials are concentrated in one place, the other place is empty, resulting in the electron's passage being cut off. Therefore, it is important that conductive polymers spread without aggregation to form a uniform network [34]. A cellulose material with high viscosity prevents the movement of conductive nanoparticles inside the cellulosic structure and helps dispersion [35], thus making nanoparticles to form a uniform electrical network [34]. CMC-PANI showed more than 20 times less viscosity than MC-PANI or HPMC-PANI. This could explain the low electrical conductivity of CMC-PANI.

The article "Development of cellulose-based conductive fabrics with electrical conductivity and flexibility" was published in 2020. Journal: PLoS One.

### Flexibility and crease recovery

Fig 4 indicates the results of the flexibility of BC-PANI and CC-PANI based on the modified heart-loop method. A sample has good flexibility and dimensional stability when it has circular shaped loop and is easily returned to its original shape [36]. As shown in Fig 4, a difference in the flexibility was observed in each sample. First, in BC and BC-PANI samples, angular shaped loops were formed rather than circular shaped ones that were formed in chemical celluloses such as MC, HPMC, and CMC. Moreover, after 1 minute of making loops, BC and BC-PANI maintained the folded shape and did not return to their original state. Based on these results, it was confirmed that the flexibility of BC and BC-PANI was relatively lower than chemical celluloses. MC and MC-PANI samples formed circular loops and returned to their original state without causing a deformation. CMC, HPMC, and HPMC-PANI samples also formed round shaped loops and displayed a tendency to retain their original states. However, fabric deformation was observed in those samples and CMC-PANI was fractured due to its low flexibility.

**Fig 4:** Flexibility of BC-PANI, MC-PANI, HPMC-PANI, and CMC-PANI.

In order to verify the flexibility test results with quantitative measurements, crease recovery test was conducted (Table 4). The highest crease recovery value was obtained at MC-PANI with 100% of crease resistance. High crease recovery angle stands for good crease recovery of the sample. Thus, the crease recovery test result indicated that MC had relatively good crease recovery after the polymerization of PANI. From these results, it was observed that MC-PANI had the highest flexibility compared to other samples such as BC-PANI, HPMC-PANI, and CMC-PANI.

The article "Development of cellulose-based conductive fabrics with electrical conductivity and flexibility" was published in 2020. Journal: PLoS One.

**Table 4:** Crease recovery of BC-PANI and CC-PANI (polymerization conditions for BC-PANI: pH level of DBSA solution = 2.0, DBSA:aniline:APS = 1:1:1, 20°C, 3 h, polymerization conditions for CC-PANI: pH level of DBSA solution = 2.0, DBSA:aniline:APS = 1:1:1, 4°C, 2 h).

	Crease recovery (%)
BC-PANI	25
MC-PANI	100
HPMC-PANI	86
CMC-PANI	N/A

### Chemical structures

The chemical structures of BC-PANI and CC-PANI were evaluated by FT-IR spectroscopy (Fig 5). The IR spectra of BC-PANI and CC-PANI showed peaks indicating the presence of cellulose (Table 5). The peaks ranging from 3340 cm^-1^ to 3450 cm^-1^ were due to the stretching vibration of hydroxyl groups [37]. The peaks near 2900 cm^-1^ were due to the asymmetric stretching vibration of the C—H bonds in cellulose [38–40]. Particularly, in the spectrum of CMC-PANI, a peak that appeared at 1589 cm^-1^ was ascribed to the carboxyl groups in CMC [41]. These peaks confirmed that BC and CC maintained cellulose structures after PANI was polymerized.

**Fig 5:** FT-IR spectra of (A) pure BC, and pure MC, (B) BC-PANI, and MC-PANI, (C) pure HPMC, and pure CMC, and (D) HPMC-PANI, and CMC-PANI (polymerization conditions for BC-PANI: pH level of DBSA solution = 2.0, DBSA:aniline:APS = 1:1:1, 20°C, 3 h, polymerization conditions for CC-PANI: pH level of DBSA solution = 2.0, DBSA:aniline:APS = 1:1:1, 4°C, 2 h).

**Table 5:** Characteristic peaks of cellulose in the FT-IR spectra of pure BC, pure MC, pure HPMC, and pure CMC.

Wavenumber (cm^-1^)					Peak assignment
Peak no.	BC	MC	HPMC	CMC	
1	3342	3450	3480	3332	O—H stretching [37]
2	2895	2894	2904	2914	C—H stretching [38–40]
		2829	2837		
3				1589	COO^—^asymmetric stretching [41]

In addition, characteristic peaks of PANI were observed in the IR spectra of BC-PANI and CC-PANI (Table 6). The original O—H stretching vibration peaks were shifted to 3240 cm^-1^ to 3230 cm^-1^ because of the N—H stretching of PANI [42]. The absorption peaks at 1612 cm^-1^ to 1606 cm^-1^ were ascribed to the C〓N stretching of quinoid ring [42–44]. The peaks at 1436 cm^-1^ to 1411 cm^-1^ were assigned to the C〓C stretching of quinoid ring [43, 45–48]. The peaks at 1315 cm^-1^ to 1307 cm^-1^ confirmed the protonated state of PANI with C—N stretching [46–50]. The results confirmed that PANI was successfully polymerized while maintaining the cellulose structures of BC and CC.

The article "Development of cellulose-based conductive fabrics with electrical conductivity and flexibility" was published in 2020. Journal: PLoS One.

**Table 6:** Characteristic peaks of PANI in the FT-IR spectra of BC-PANI and CC-PANI (polymerization conditions for BC-PANI: pH level of DBSA solution = 2.0, DBSA:aniline:APS = 1:1:1, 20°C, 3 h, polymerization conditions for CC-PANI: pH level of DBSA solution = 2.0, DBSA:aniline:APS = 1:1:1, 4°C, 2 h).

Wavenumber (cm^-1^)					Peak assignment
Peak no.	BC-PANI	MC-PANI	HPMC-PANI	CMC-PANI	
1	3240	3282	3230	3232	N—H stretching [42]
2	1612	1606	1606		C〓N stretching of quinoid ring [42, 44]
3		1568	1567	1571	C〓C stretching of benzenoid ring [45–48]
4	1425	1436	1423	1411	C〓C stretching of quinoid ring [43, 45–48]
5	1313	1307	1309	1313	C—N stretching of secondary amine [46–50]

### Crystalline structures

XRD was used to characterize the crystalline structure of BC-PANI and CC-PANI. Both BC-PANI and CC-PANI showed reflection peaks characteristic of a cellulose structure (Fig 6). The cellulose peaks were observed at 14.7° and 22.8° for BC-PANI [51] and 7.91° and 20.53° for MC-PANI [38, 52], 8.87° and 19.88° for HPMC-PANI, and 8.87° and 20.62° for CMC-PANI [53, 54]. This suggested that cellulose structures of both BC and CC remained after the polymerization of PANI.

**Fig 6:** XRD patterns of (A) pure BC and BC-PANI, (B) pure MC pure and MC-PANI, (C) pure HPMC and HPMC-PANI, and (D) pure CMC and CMC-PANI (polymerization conditions for BC-PANI: pH level of DBSA solution = 2.0, DBSA:aniline:APS = 1:1:1, 20°C, 3 h, polymerization conditions for CC-PANI: pH level of DBSA solution = 2.0, DBSA:aniline:APS = 1:1:1, 4°C, 2 h).

Characteristic peaks of PANI were also appeared in the XRD patterns of both BC-PANI and CC-PANI. For BC-PANI, the peak at 23.7° indicated that PANI inside BC was partially crystalline [55], and the peak at 26.7° was attributed to the parallel arrangement of PANI polymer chains [56]. For CC-PANI, the broad peak around at 20.26° was ascribed to the presence of the emeraldine state of PANI with good electrical conductivity [46–48]. There were more peaks at 23.46° and 25.19° for HPMC-PANI, 23.5° and 25.46° for CMC-PANI, respectively, which are assembled peaks in XRD data of PANI [57]. The peak at 28.57° appeared in CMC-PANI was attributed to the periodicity perpendicular to the PANI chain direction [58]. These peaks demonstrated that PANI was successfully polymerized inside BC-PANI and CC-PANI.

Data on the degree of crystallinity of BC-PANI and CC-PANI, and the percent change before and after the polymerization of PANI are presented in Table 7. As shown in Table 7, the crystallinity of BC-PANI, MC-PANI, ad HPMC-PANI were decreased by 19.1%, 21.8%, and 34.1%, respectively, whereas that of CMC-PANI was increased by 46.7%. This can be explained by the amorphous nature of PANI polymer. PANI has low crystallinity due to the repetitive formation of benzenoid and quinoid rings in PANI chains [59]. Thus, it is confirmed that the degree of crystallinity decreases as the cellulosic structure effectively anchors the PANI molecules. It can also explain why CMC-PANI exhibited the lowest electrical conductivity among the four conductive cellulose fabrics.

The article "Development of cellulose-based conductive fabrics with electrical conductivity and flexibility" was published in 2020. Journal: PLoS One.

**Table 7:** Crystallinity degrees of BC-PANI and CC-PANI (polymerization conditions for BC-PANI: pH level of DBSA solution = 2.0, DBSA:aniline:APS = 1:1:1, 20°C, 3 h, polymerization conditions for CC-PANI: pH level of DBSA solution = 2.0, DBSA:aniline:APS = 1:1:1, 4°C, 2 h).

	Crystallinity (%)		Percent change (%)
	Before polymerization	After polymerization	
BC-PANI	77.4	65.0	-19.1
MC-PANI	60.9	50.0	-21.8
HPMC-PANI	52.7	39.3	-34.1
CMC-PANI	32.8	61.5	46.7

### Surface characterization

The surface morphologies of BC-PANI and CC-PANI were examined by SEM. Fig 7(A) shows the fibrous network structure of pure BC. A three-dimensional nanostructure built from cellulose nanofibers was clearly observed. In the SEM image of BC-PANI (Fig 7(B)), the BC fibers appeared thicker than those in the pure BC, due to the coating of PANI [60]. The images confirmed that BC was polymerized with PANI without significant changes in its fibrous structure. Before observing the surface morphology of CC-PANI, the morphology of a PANI solution diluted 500-fold with isopropanol and dried on a plastic film was examined (Fig 7(C)). The polymerized PANI particles were in spherical structures that were approximately 10 to 30 nm in diameter. This was due to the emulsion polymerization, since the size and shape of PANI particles corresponded to those of micelles [61]. Unlike pure BC, pure CC (Fig 7(E), 7(G) and 7(I)) did not show a fibrillar structure, but rather had a sheet type plane structure [62, 63]. Notably, in the SEM images of CC-PANI (Fig 7(D)), coagulated spherical structures were observed on the surface of CC, indicating the presence of PANI. The findings might reflect the influence of the spreading coefficient of the solvent used to prepare the PANI solution.

**Fig 7:** SEM images of (A) BC, (B) BC-PANI (C) emulsion polymerized PANI, (D) MC-PANI with same magnitude with (C), (E) MC, (F) MC-PANI, (G) HPMC, (H) HPMC-PANI, (I) CMC, (J) CMC-PANI with scale bars provided in the images. (polymerization conditions for BC-PANI: pH level of DBSA solution = 2.0, DBSA:aniline:APS = 1:1:1, 20°C, 3 h, polymerization conditions for CC-PANI: pH level of DBSA solution = 2.0, DBSA:aniline:APS = 1:1:1, 4°C, 2 h).

## Discussion

In this study, we produced BC-PANI and CC-PANI composites with good electrical conductivity by using PANI in the emeraldine-salt state. Interestingly, we directly fabricated BC-PANI and CC-PANI by mixing BC and CC powders with a PANI solution. Importantly, it was confirmed that polymerization of PANI on MC enables the fabrication of conductive cellulose with improved electrical conductivity than BC. The findings support the view that the MC-PANI is a good conductive fabric that could potentially be used in wearable devices and sensors.
